# Evaluation of High Yielding Maize Hybrids Based on Combined Stability Analysis, Sustainability Index, and GGE Biplot

**DOI:** 10.1155/2022/3963850

**Published:** 2022-07-25

**Authors:** Dedi Ruswandi, Muhammad Syafii, Noladhi Wicaksana, Haris Maulana, Mira Ariyanti, Nyimas Poppy Indriani, Edy Suryadi, Jajang Supriatna, Yuyun Yuwariah

**Affiliations:** ^1^Faculty of Agriculture, University of Padjadjaran, Jl. Raya Bandung-Sumedang, Jatinangor, Km. 21, 45353, Indonesia; ^2^Faculty of Agriculture, University of Singaperbangsa Karawang, Indonesia; ^3^Faculty of Animal Husbandry, University of Padjadjaran, Indonesia; ^4^Faculty of Agroindustrial Technology, Universitas Padjadjaran, Bandung, Indonesia; ^5^Faculty of Agriculture, Universitas Islam Negeri Sunan Gunung Djati Bandung, Indonesia

## Abstract

Selection of high yielding and stable maize hybrid requires effective method of evaluation. Multienvironment evaluation is a critical step in plant breeding programs that is aimed at selecting the ideal genotype in a wide range of environments. A method of evaluation that combines a variety parameter of stability could provide more accurate information to select the ideal genotype. The aims of the study were (i) to identify the effect of genotype, environment, and genotype × environment interactions (GEIs) on maize hybrid yields and (ii) to select and to compare maize hybrids that have high and stable yields in diverse environments in Sumatra Island based on combined analysis, selection index, and GGE biplot. The study was conducted in five different environments in Sumatra Island, Indonesia, using a randomized complete block design repeated three times. Data were estimated using combined variance analysis, parametric and nonparametric stability, sustainability index, and GGE biplot. The results showed that the genotype had a significant effect on maize hybrid yields with a contribution of 41.797%. The environment contributed to 24.314%, and GEIs contributed 33.889% of the total variation. E1 (Karo, South Sumatra; dry season) and E3 (Tanjung Bintang, Lampung; dry season) were identified as the most ideal environments (representative) for testing the hybrids for wider adaptability. The maize hybrid with high and stable yields can be selected based on combined stability analysis and sustainability index as well as GGE biplot. These three methods are effectively selected high yielding and stable genotypes when they are used together. The three maize hybrids, namely, MH2, MH8, and MH9, are recommended as high yielding and stable genotype candidates.

## 1. Introduction

Indonesia is the major maize producer in South East-Asian (SEA) region and also among the main maize producer countries in the world. In 2021, Indonesia produced more than 20 million tons of maize grain [1]. Sumatra Island is one of the main maize producers in Indonesia. Among the main maize producers in Sumatra Island are Lampung and North Sumatra. Lampung places third in Indonesia with a harvested area of 474 900 ha and production of 2.83 million tons of maize while North Sumatra ranks fourth highest in Indonesia with a harvested area of 350 600 ha and produces 1.83 million tons [2]. Based on this data, evaluation of new maize hybrids from the Sumatra Island is a must to increase maize production in Indonesia and the SEA region.

Multienvironment evaluation is important since it can determine genotype × environment interactions (GEIs). Through the multienvironment evaluation, high yielding and stable maize hybrids can be selected. The occurrence of GEIs, however, indicated that various genotypes can have different responses to environmental changes and make the selection process inefficient [3–5]. In some cases, maize yields are strongly influenced by GEIs due to environmental changes [5–8]. Studies also reported that GEIs complicate the selection process for crops like sweet potato in Indonesia [9], durum wheat in Turkey [10], yellow passion fruit in Brazil [11], and cotton in China [12]. Therefore, GEI analysis is important in evaluating superior genotypes.

The formation of stable and high yielding maize hybrids in accordance with consumer preferences is the main objective of maize plant breeding programs. To achieve this, multienvironment evaluation is important. It helps determine stable genotypes in a wide range of environments that are also adaptive to a specific environments. The effect of GEIs on multienvironment evaluation mainly occurs using quantitative characters including grain yields [8] as well as resistance to biotic and abiotic factors [13].

Selection of stable and high-yielding genotypes can combine parametric and nonparametric stability models. This method has been applied in selecting high yielding and stable genotypes of many crops including in chickpeas [14], grass bean [15], wheat [16], barley [17, 18], sweet potato [9], and peanut [19]. The use of combined analysis of the various stability parameters together with the multivariate GGE biplot for selecting stable and high yielding genotypes in multienvironment evaluation is recommended. The advantages of these approaches in selection of stable varieties for different environments and specific varieties in specific environments were described by [18] as follows: (i) the parametric stability was under statistical assumptions such as interaction effects and normal distribution of errors; (ii) the nonparametric stability was used based on the performance of ranks of data, and no assumptions are required for distribution of model residuals and homogeneity of variances [20]; (iii) the GGE biplot was used to determine the pattern of genotypic responses across environments in multienvironments evaluation [21]. The objectives of the study were (i) to identify the effect of genotype, environment, and genotype × environment interactions (GEIs) on maize hybrid yields and (ii) to select and to compare maize hybrids that have high and stable yields in diverse environments in Sumatra Island based on combined analysis, selection index, and GGE biplot.

## 2. Material and Methods

### 2.1. Plant Materials

The genetic materials used included seven new maize hybrids and four commercial varieties as checks (Table 1). These genotypes were the result of plant breeding program developed by the Faculty of Agriculture, Universitas Padjadjaran (UNPAD). The new maize hybrids had different genetic backgrounds [22].

### 2.2. Field Experiments and Data Collection

Field experiments were conducted in five environments in the Sumatra Island, Indonesia, namely, Karo (North Sumatra; dry season 2018) (E1), Karo (North Sumatra; rainy season 2018/2019) (E2), Tanjung Bintang (Lampung; dry season 2018) (E3), Gunung Sugih (Lampung; rainy season 2018/2019) (E4), and Gunung Sugih (Lampung; dry season 2020) (E5). These locations are main producer of maize in Sumatera Island. The experiment was designed in a randomized complete block design which was repeated three times. Each hybrid was planted in four rows plot, 5 m long and at a spacing of 0.75 × 0.25 m. The data were gathered at harvest following the standard descriptor for maize [23]. The yield of each hybrid in each experimental plot was converted in ton. ha^−1^.

### 2.3. Data Analysis

The combined ANOVA statistical model to estimate GEIs follows the equation:

(1) $$\begin{array}{c} Y_{opqr}=\mu +G_{o}+E_{p}+{GE}_{op}+R_{q\left(p\right)}+B_{r\left(q\right)}+\varepsilon_{opqr,} \end{array}$$

where *Y*_*opqr*_ is the value of maize hybrid *o* in plot *r* and the value in environment *p* of each replication *q*, *μ* is the grand mean of grain yield, *G*_*o*_ is the effect of maize hybrid *o*, *E*_*p*_ is the effect of the environment *p*, *GE*_*op*_ is the effect of GEIs on maize hybrid *o* and environment *p*, *R*_*q*(*p*)_ is the effect of replicate *q* on environment *p*, *B*_*r*(*q*)_ is the effect of replication *q* on plot *r*, and *ε*_*opqr*_ is the error effects from maize hybrid *o* in plot *r* and repeat *q* of environment *p*, respectively. The combined ANOVA was calculated using GenStat 12th. If the data shows that GEIs have a significant effect, then the yield stability analysis is carried out using parametric and nonparametric stability, sustainability index (SI), and GGE biplot.

Nonparametric and parametric stability models were used to identify stable and high yield maize hybrids. Parametric stability linear regression (*b*_*i*_) is measured followed [24]. According to [24], a genotype was declared stable if it has a regression deviation = 1, and the variance deviation value (*S*^2^di) = 0. To estimate mean variance component (*θ*_*i*_), following [25] with the formula:

(2) $$\begin{array}{c} \theta_{i}=\frac{p}{2\left(p-1\right)\left(q-1\right)}\overset{q}{\underset{j-1}{\sum }}{\left(x_{ij}-{\bar{X}}_{i.}+{\bar{X}}_{.j}+{\bar{X}}_{\cdots }\right)}^{2}+\frac{SSGE}{2\left(p-2\right)\left(q-1\right)}. \end{array}$$

GE variance component (*θ*_(*i*)_), this parameter was calculated as follows [26]:

(3) $$\begin{array}{c} \theta_{\left(i\right)}=\frac{-p}{\left(p-1\right)\left(p-2\right)\left(q-1\right)}\overset{q}{\underset{j-1}{\sum }}{\left(x_{ij}-{\bar{X}}_{i.}-{\bar{X}}_{.j}+{\bar{X}}_{..}\right)}^{2}+\frac{SSGE}{\left(p-2\right)\left(q-1\right)}. \end{array}$$

Wricke's ecovalence (W_*i*_^2^) was estimated as follows [27]:

(4) $$\begin{array}{c} {\text{W}}_{i}^{2}=\sum {\left(X_{ij}-{\bar{X}}_{i.}-{\bar{X}}_{.j}+{\bar{X}}_{..}\right)}^{2}. \end{array}$$

Shukla's stability variance (*σ*_*i*_^2^) for the genotype *i* was measured as follows [28]:

(5) $$\begin{array}{c} \sigma_{i}^{2}=\left|\frac{p}{\left(p-2\right)\left(q-1\right)}\right|{\text{W}}_{i}^{2}-\frac{\sum W_{i}^{2}}{\left(p-1\right)\left(p-2\right)\left(q-1\right)}. \end{array}$$

Coefficient of variance (CV_*i*_) was followed [29] with the formula:

(6) $$\begin{array}{c} {\text{CV}}_{i}=\frac{{\text{SD}}_{g}}{\bar{X}}\times 100. \end{array}$$

For all parameters used, *x*_*ij*_ is the grand grain yield from the maize hybrid*i*across all sites, ${\bar{X}}_{i.}$ is the mean of grain yield from maize hybrid *i*, ${\bar{X}}_{.j}$ is the mean of grain yield in site *j*, ${\bar{X}}_{..}$is the overall average grain yield, *p* and *q* are the numbers of maize hybrid and environment, and SD_g_ is the standard deviation of a GEIs.

Nonparametric stability (*S*^(*i*)^) measures following [20, 30] with the formula as follows:

(7) $$\begin{array}{c} S_{i}^{\left(1\right)}=2\overset{n-1}{\underset{j}{\sum }}\frac{\sum_{j\prime =j+1}^{n}\left|r_{ij}-r_{ij}^{\prime }\right|}{\left[N\left(n-1\right)\right]},\\ S_{i}^{\left(2\right)}=\frac{\sum_{j=1}^{n}{\left(r_{ij}-{\bar{r}}_{i.}\right)}^{2}}{\left(N-1\right)},\\ S_{i}^{\left(3\right)}=\frac{\sum_{j=1}^{n}{\left(r_{ij}-{\bar{r}}_{i.}\right)}^{2}}{{\bar{r}}_{i}},\\ S_{i}^{\left(6\right)}=\frac{\sum_{j=1}^{n}\left|r_{ij}-{\bar{r}}_{i.}\right|}{{\bar{r}}_{i.}}, \end{array}$$

where *r*_*ij*_ is the rank of stability from maize hybrid *i* in the environment *j*, ${\bar{r}}_{i.}$ is the mean rank across all environment for each maize hybrid, and *N* is the number of environment. Parametric stability (NP^(*i*)^) measures following [31] with the formula as follows:

(8) $$\begin{array}{c} {\text{NP}}^{\left(1\right)}=\frac{\sum_{j=1}^{n}\left|r_{ij}^{*}-M_{di}^{*}\right|}{N},\\ {\text{NP}}^{\left(2\right)}=\frac{\left[\sum_{j=1}^{n}\left|r_{ij}^{*}-M_{di}^{*}\right|/M_{di}\right]}{N},\\ {\text{NP}}^{\left(3\right)}=\frac{\sqrt{\sum {\left(r_{ij}^{*}-r_{i.}^{*}\right)}^{2}/N}}{{\bar{r}}_{i.}},\\ {\text{NP}}^{\left(6\right)}=\frac{2x\left[\sum_{j=1}^{n-1}\sum_{j^{\prime }=j+1}^{n}\left|r_{ij}^{*}-r_{i.}^{*}\right|/{\bar{r}}_{i.}\right]}{N\left(\text{N}-1\right)}, \end{array}$$

where *r*_*ij*_^∗^ is the stability rank in environment *j* from maize hybrid *i* based on adjusted data, *M*_*di*_^∗^ is the median rank for adjusted data (grain yield), *M*_*di*_ is the original data from the same parameters, and *N* is the number of environment. Kang rank's (KR) nonparametric stability model is followed formula by [32]. In this method, grain yield performance and stability variance that identify high yielding and stable genotypes are given a weighting value of 1. The stable genotypes were identified based on nonparametric and parametric stability measurements using STABILITYSOFT (online software) [33]. To select and to compare high yield maize hybrids based on combined analysis, the results of parametric and nonparametric stability were grouped using cluster analysis (dendrogram) based on the stability rank of each parameter. Cluster analysis was estimated using the SPSS v19 software [34].

The sustainability index (SI) was estimated by the following formula [35]:

(9) $$\begin{array}{c} \text{SI}=\left[\frac{\left(Y-\sigma \text{n}\right)}{\text{YM}}\right]\times 100, \end{array}$$

where *Y* is the mean performance of a maize hybrid, *σn* is the standard deviation, and YM is the best performance of a maize hybrid in any environment. The SI values were classified arbitrarily into five groups, i.e., very low (up to 20%), low (21% to 40%), moderate (41% to 60%), high (61% to 80%), and very high (above 80%) [36]. SI was calculated using MS Excel 2013.

To select and compare the stability and adaptability of maize yield based on GGE biplot, the model for GGE biplot was followed [37] with the formula:

(10) $$\begin{array}{c} \;{Ῡ}_{mn}-\mu_{m}=\beta_{n}+\sum_{k=1}^{t}\lambda_{o}\alpha_{mo}\gamma_{no}+\varepsilon_{mn}, \end{array}$$

where *Ῡ*_*mn*_, *μ*_*m*_, *β*_*n*_, *k*, *λ*_*o*_, *α*_*mo*_ and *γ*_*no*_, and *ε*_*mn*_ are the performance in location “*n*” from maize hybrid “*m*,” overall average yield, the influence of location “*n*,” number of primer components, the singular value from primer component “*o*,” value of maize hybrid “m” and location “n” for primer component “*o*,” and the error of the maize hybrid “*m*” in location “*n*,” respectively.

## 3. Results and Discussions

### 3.1. Genotype by Environment Interactions (GEIs) of Maize Hybrids in Sumatra Island

The combined analysis of variance (ANOVA) for yield of maize hybrids in five environments in the Sumatra Island is presented in Table 2. The genotypes, environments, and their interactions (GEIs) have a significant effect on maize yields with contributions of 41.797%, 24.314%, and 33.889%, respectively.

The genotype effects provided the highest contribution to the grain yield variation. The high “sum of square (SS)” value of the genotypic effect was due to the highly variable yield performance of the hybrids. The smaller value of GEIs compared to the genotype effect implies that the stable genotypes across environments and the maximum variation in hybrid performance were contributed by genetic variance. The high genotype differences in this analysis may be due to the fact that the material used is a new hybrid that has not yet been released nationally thus requiring extensive testing in multienvironments. Ruswandi et al. [38] also revealed that the differences in genotypes can cause grain yield variations in multienvironment trials. In another study, Karuniawan et al. [39] reported that differences in the origin of the genotypes used can also be a differentiator for potential yields. In addition, the environmental factors such as locations, seasons, and cultivation systems also have a significant influence which means that the conditions of the planting affected yield performances [36]. The percentage of environmental influence which is quite large on grain yields indicates that the selected environment is quite diverse. Differences in environmental conditions during planting can lead to differences in yield and yield quality of maize hybrid [6, 8, 40]. The response of maize hybrids to the tested environment is the variable indicated by the GEIs. The GEI effect also has implications in the plant selection process. The emergence of GEIs can make the selection process difficult and inefficient [5, 38, 41]. The emergence of GEIs in multienvironment evaluation requires stability analysis to select high yielding and stable genotypes in a wide range of environment.

### 3.2. Evaluation of High Yielding Maize Hybrids Using Combined Stability Analysis

Stability parameter(s) has been widely used by plant breeders to select high yielding and stable genotype(s). Various methods have been proposed to estimate stability parameters [9, 14, 16–18]. In this study, several parametric and nonparametric stability parameters and sustainability index (SI), as well as the GGE biplot model, were estimated and were compared to identify high yielding and stable maize hybrids.

Stability parameters of maize hybrids and their ranks based on parametric and nonparametric estimation are presented in Table 3. All nonparametric stability parameters select MH2 as the most stable hybrid. On the other hand, several stability parameters, including W*i*^2^, *σ*_*i*_^2^, *s*^2^*d*_*i*_, Cvi, and *θ*_(*i*)_, which are estimated using parametric method of stability indicated MH2 as the most stable, while other parametric stability parameters determined different genotypes such as MH5 by stability parameter of bi and MH6 by stability parameter of *θ*_(*i*)_. In the parametric method of stability analysis, there were stability parameters that have similar stability rank (correlation = 1), namely, Wricke equivalence (W_*i*_^2^), Shukla stability variance (*σ*_*i*_^2^), and GE Plaisted variance component (*θ*_(*i*)_) which selected MH2 as the most stable hybrid followed by MH9 and MH5. Similar results were also shown by [42], which reported that the three stability parameters (W_*i*_^2^, *σ*_*i*_^2^, *θ*_(*i*)_) gave similar rank of stability during evaluation of sweet potato yields in Indonesia. This indicated that the three parameters (W_*i*_^2^, *σ*_*i*_^2^, *θ*_(*i*)_) have the same power in estimating genotype stability; therefore, the three stability parameters were suggested to select stable genotypes [9, 18]. Based on the average ranks (AR), the maize hybrid of MH2 followed by MH8, MH9, and MH5 had a small AR value; therefore, these maize hybrids can be proposed as the most stable genotype. MH4 maize hybrid followed by MH6 and MH11 had the largest AR value; hence, they are the most unstable genotypes. Vaezi et al. [18] stated that the genotype with the lowest AR value has the highest yield stability in multienvironment evaluation. Thus, genotypes that have a small AR value were more desirable. To select and to compare high yield maize hybrids, the results of parametric and nonparametric stability were grouped using a hierarchical cluster analysis (HCA) based on the stability rank of each parameter.

The results of the HCA are presented in Figure 1. The dendrogram separated the maize hybrid genotypes into four main groups. The first group consisted of MH5 and MH10 genotypes. This group has a medium average yield and low AR, so they were stable genotypes with medium yields. This group can be an alternatives, because they have grain yields that are in the range between low and high. The second group consisting of MH2, MH8, and MH9 had an average yield above the overall average yield with a low AR value. All three genotypes belong to the ideal group because they have high and stable yields in five experimental environments. Several researchers have also succeeded in selecting high yielding and stable genotypes by parametric and nonparametric stability parameters, including in barley [17], soybean [43], wheat [18], and sweet potato [39]. The genotypes in the second group, therefore, can be recommended as new superior genotypes that are stable and high yielding. This ideal group is expected to support the development of new varieties. The third group consisted of MH4, MH7, and MH11 genotypes. This group has low yields but high AR values, so it belongs to the unstable low yield group. The genotypes in this group were less desirable because they will be difficult to use for sustainable variety development programs. The fourth group consisted of MH1, MH3, and MH6 genotypes. This group has a high AR value but has a high average yield. These genotypes are included in the unstable high yield group (specific adapted). The specific adapted genotypes have an advantage in response to environmental changes compared to stable genotypes [44–46]. Therefore, this group can be recommended as specific adapted high yielding genotypes.

### 3.3. Evaluation of High Yielding Maize Hybrids Based on Sustainability Index (SI)

The results of sustainability index (SI) analysis is presented in Table 4. According to researchers a high SI value indicated the stability levels of a genotype [35, 36, 47]. The distribution of SI values was based on the opinion of [36] which stated that SI values are divided into five groups, namely, very low, low, medium, high, and very high. The estimated SI value of maize yields was in the range of 47.226% (moderate) to 82.273% (very high). The moderate SI values were shown by the maize hybrids of MH4 (47.226%) and MH11 (55.101%). High SI values were possessed by maize hybrids of MH1, MH3, MH5, MH6, MH7, MH8, MH9, and MH10, whereas maize hybrid of MH2 showed the highest SI (82.273%).

Estimated analysis of variance in the SI for maize hybrid yields revealed significant differences in different environments and indicated genetic variability in the genotypes studied. The MH2 genotype recorded an average yield of 9.346 t. ha^−1^ with a very high SI of 82.273%. This indicated the best performance for this genotype (Table 4). The best performance with a high SI value can be considered as an indication of the closeness between the best performance and the average performance [48]. The next genotypes with high yields and SI values close to 80% were MH8 (9.904 t/ha with SI = 79.804%), MH10 (8.745 t/ha with SI = 77.833), MH9 (9.480 t/ha with SI = 74.191%), and MH3 (9.852 with SI = 73.159%). Several other genotypes, namely, MH1 had a high average yield (9.264 t/ha; more than the overall average) but had an SI value = 69.696%, MH5 had a low average yield (8.510) with an SI value = 71.620%, and MH7 had a low average yield (6.959) with SI value = 70.558%, indicating that the genotypes' performance was inconsistent in different environments or could provide better yield performance under favorable environmental conditions, while the other two genotypes (MH4 and MH11) showed poor yield performance and adaptability. This estimation of SI for maize hybrids was also in line with the results of combined stability analysis in Figure 1, which grouped them in the unstable low yield. In general, genotypes with high and very high SI criteria with yields above the overall average yield indicated that these genotypes belonged to the ideal group (having high and stable yield). Similar result was also reported by [47] who succeeded in selecting high yielding and stable rice using SI. Thus, these results prove that SI can be used to determine stable and high yield maize hybrids.

### 3.4. Selection of Maize Hybrid Using GGE Biplot Analysis

Visualization of yield stability of maize hybrid genotypes was estimated using GGE biplot analysis. The results of the GGE biplot analysis showed that PC1 and PC2 accounted for 50.00 and 23.63% of the total variation in maize hybrid yields, respectively (Figure 2). According to the representative vs. discriminative view of the GGE biplot (Figure 2), the test environments have the different vector length. The five environments showed significant variations and provided different conditions of grain yields of the maize hybrid. The environmental differences are depicted as vector lines originating from the biplot origin [40, 49]. The angle between the vectors of two environments indicates the correlation between them. In the biplot, the vectors E1 and E3 form an acute angle which indicates the close relationship between the two environments (Figure 2). On the other hand, E4 and E5 are negatively correlated with E2. However, both E1 and E3 have weak correlations with E2, E4, and E5. The distance between the two environments showed their dissimilarity in differentiating genotypes, and the close relationship between the test environments indicates that the same information can be obtained from fewer environments which can reduce testing costs. Therefore, one test site could be dropped in this case.

The experimental environment in the GGE biplot was categorized into three types, namely, the class I environment which has a short vector and shows limited information about the genotype, so it must be rejected as a test environment; class II produces extended vectors and low angles of view with an abscissa environmental mean coordinate, so they are the best models for selecting the best genotypes; and class III has long vectors and produces a sufficiently large angle with an average of the environmental coordinates of the abscissa; therefore, they should reject a perfect genotype assessment, but it can be used in selecting adaptive genotypes [49]. The results of the GGE biplot measurement showed that the E5 is included in class I because it has the shortest vector, so it is not suitable as a test environment. Environments that are included in class II were E3 and E1, while other environments were included in class III. In Figure 3 (environment rank), the ranking of each environment was indicated by how close the environmental point was to the ideal point (small arrow). According to Ruswandi et al. [8], the ideal environment was the environment that has the closest distance to the ideal point. In our study on the Sumatra Island, the E3 shows the position closest to the ideal point, followed by E1, while the other environment was outside the circle and has a large enough angle with the ideal point. This indicates that the E3 was the most ideal environment in selecting stable and high yielding genotypes, while other environments can be used to select adaptive genotypes.

The “which won where” pattern indicated that the five locations have five sectors with different peak genotypes (Figure 4). The environments that are in the same sector are the locations that have the best genotypes and are considered as megaenvironments (MEs) for that genotype [40]. There were three sectors containing the environment, namely, sector 1 contained the E2 environment with a peak genotype of MH6, sector 2 contained E1 and E3 (MEs1) with a peak genotype of MH8, and sector 3 contained E4 and E5 (MEs2) with a peak genotype of MH3. Genotypes that are at the top of each sector have high yields in the environment in that sector [46, 50, 51]. Genotypes that are in sectors contained more than one environment or megaenvironment and show an ideal genotype [52–54]. Therefore, in this study, the ideal genotypes were MH2, MH8, MH9, MH1, MH3, and MH10. The test results also showed that the peak genotypes located in sectors that do not contain the environment have low grain yields in all environments, so the genotypes in this sector are not recommended for development programs.

The results of the GGE biplot analysis showed that several identified genotypes were close to the center of the axis (Figure 4). The genotypes were MH5 and MH10. Several researchers revealed that genotypes that were close to the central axis (0.00) were stable genotypes [46, 51]. However, stability must be classified by yield performance. To determine the genotypic stability ranking based on the GGE biplot, the “mean vs. stability” pattern was used (Figure 5). Based on Figure 5, the ideal genotype was the closest to the stability line and the ideal point (small arrow) [8, 55]. Based on this pattern, MH8, MH9, and MH2 were closest to the ideal line and point (small arrow). Therefore, all three genotypes were considered as ideal genotypes. The results of the combined stability analysis, sustainability index (SI), and GGE biplot showed a similar pattern in selecting the ideal genotype (stable and high yielding). The combined stability analysis selected MH2, MH8, and MH9 as the high yielding and stable genotypes. The sustainability index (SI) selected MH2, MH8, MH10, MH9, and MH3 as the best genotypes, while the GGE biplot selected MH2, MH8, and MH9 as the best genotypes. Based on the combined stability measurements, three ideal maize hybrid genotypes were selected in five test environments, namely, the MH2, MH8, and MH9 genotypes. These three genotypes can be recommended as new superior genotypes that were stable and high yielding in the Sumatra Island and as plant material for the next maize plant breeding program.

## 4. Conclusion

Genotype, environments, and GEIs have a significant effect on maize hybrid yields with a contribution of 41.797%, 24.314%, and 33.889% of the total variation, respectively. E1 and E3 were identified as the most ideal environments (representative) for testing the hybrids for wider adaptability. MH2, MH8, and MH9 were selected as genotypes with high and stable yields. These three genotypes can be recommended as candidates for new superior genotypes that are stable and high yielding. In addition, combined stability analysis, sustainability index, and GGE biplot were effective for selection of high and stable maize hybrids.

## Figures and Tables

**Figure 1:** Combined stability analysis of maize hybrids using a hierarchical cluster analysis (HCA) based on the stability rank of each stability parameter.

**Figure 2:** GGE biplot “discrimination vs. representativeness” on maize hybrids in five environments. E1: Karo (South Sumatra; dry season); E2: Karo (South Sumatra; rainy season); E3: Tanjung Bintang (Lampung; dry season); E4: Gunung Sugih (Lampung; rainy season); E5: Gunung Sugih (Lampung; dry season).

**Figure 3:** GGE biplot “ranking environments” on maize hybrids in five environments. E1: Karo (South Sumatra; dry season); E2: Karo (South Sumatra; rainy season); E3: Tanjung Bintang (Lampung; dry season); E4: Gunung Sugih (Lampung; rainy season); E5: Gunung Sugih (Lampung; dry season).

**Figure 4:** GGE biplot “which, won, where/what” on maize hybrids in five environments. E1: Karo (South Sumatra; dry season); E2: Karo (South Sumatra; rainy season); E3: Tanjung Bintang (Lampung; dry season); E4: Gunung Sugih (Lampung; rainy season); E5: Gunung Sugih (Lampung; dry season).

**Figure 5:** GGE biplot “mean vs. stability” on maize hybrids in five environments. E1: Karo (South Sumatra; dry season); E2: Karo (South Sumatra; rainy season); E3: Tanjung Bintang (Lampung; dry season); E4: Gunung Sugih (Lampung; rainy season); E5: Gunung Sugih (Lampung; dry season).

**Table 1:** The maize hybrid materials used in the experiment.

Code	Hybrid	Parental line			Pedigree
		Female		Male	
MH1	Cx				Hybrid commercial of Cargill
MH2	Pxy				Hybrid commercial of Pioneer
MH3	NKxx				Hybrid commercial of Monsanto
MH4	Bisi x				Hybrid commercial of Bisi
MH5	PA	1011	×	1016	Female is a downy mildew resistant line; male is a high nutrition line
MH6	PB	1014	×	1018	Female is a downy mildew resistant line, and male is a high protein line
MH7	PC	1019	×	1020	Both parents are high nutrition lines
MH8	PE	1007	×	1008	Female is a high yield line, and male is a high nutrition line
MH9	PF	1006	×	1007	Female is a high nutrition line, and male is a high yield line
MH10	PG	1008	×	1009	Female is a high nutrition line; male is a downy mildew resistant line
MH11	PH	1002	×	1003	Female is a high nutrition and downy mildew resistant line; male is a high yield line

**Table 2:** Combined analysis of variance for grain yield.

Source	df	SS	MS	*F* value	pr (>f)		TSS explained (%)
Env	4	127.552	31.888	86.2541	1.04*E*-07	^∗∗^	24.314
Rep (env)	10	3.697	0.370				
Gen	20	219.273	10.964	20.7798	<2.2*e*-16	^∗∗^	41.797
Gen × Env	40	177.788	4.445	8.4242	<2.2*e*-16	^∗∗^	33.889
Residual	90	47.485	0.528				
Min (t.ha^−1^)	2.989						
Max (t.ha^−1^)	12.481						
Mean (t.ha^−1^)	8.719						
CV (%)	8.331						

Df: degree freedom; SS: sum of square; MS: mean of square; Env: environments; Rep: replications; Gen: genotypes; Min: minimum value; Max: maximum value; CV: coefficient of variation.

**(a):** 

Genotype	*Y*	*S* ^(1)^	*S* ^(2)^	*S* ^(3)^	*S* ^(6)^	NP^(1)^	NP^(2)^	NP^(3)^	NP^(4)^	*K*R	W_*i*_^2^	*σ*_*i*_^2^	*s* ^2^ *d*_*i*_	*b*_*i*_	CV_*i*_	*θ*_(*i*)_	*θ*_*i*_
MH1	9.264	4.000	10.700	6.294	1.941	4.000	0.320	0.534	0.588	12	5.905	1.624	0.828	0.834	15.740	1.621	1.713
MH2	9.346	1.000	0.800	0.432	0.486	1.200	0.175	0.226	0.135	5	0.753	0.050	0.098	0.871	10.212	1.778	1.004
MH3	9.851	3.800	10.300	4.905	1.619	3.000	0.236	0.430	0.452	10	6.905	1.930	0.923	0.662	14.500	1.590	1.850
MH4	7.429	2.800	8.000	10.667	3.333	3.000	2.200	1.108	0.933	19	12.218	3.553	1.094	2.082	33.337	1.428	2.581
MH5	8.510	2.600	5.300	3.786	1.714	3.000	0.400	0.497	0.464	11	1.950	0.416	0.278	0.988	14.087	1.742	1.169
MH6	9.316	4.600	14.200	8.353	2.235	4.200	0.320	0.581	0.676	16	15.656	4.604	2.062	0.440	20.920	1.323	3.053
MH7	6.959	2.400	4.300	6.615	2.923	2.600	1.467	1.088	0.923	18	6.625	1.844	0.886	0.670	20.254	1.599	1.812
MH8	9.904	2.600	4.800	2.286	0.905	2.600	0.244	0.384	0.310	6	2.985	0.732	0.412	0.838	11.961	1.710	1.311
MH9	9.480	2.800	5.200	2.537	1.073	1.600	0.200	0.236	0.341	5	1.362	0.236	0.121	1.364	14.998	1.760	1.088
MH10	8.745	3.000	6.500	4.333	1.333	2.400	0.467	0.501	0.500	11	2.374	0.545	0.337	0.931	13.688	1.729	1.227
MH11	7.107	2.400	4.200	6.000	3.143	3.800	1.240	1.298	0.857	19	8.112	2.298	1.102	1.320	26.785	1.553	2.016

**(b):** 

Rank	*Y*	*S* ^(1)^	*S* ^(2)^	*S* ^(3)^	*S* ^(6)^	NP^(1)^	NP^(2)^	NP^(3)^	NP^(4)^	*K*R	W_*i*_^2^	*σ*_*i*_^2^	*s* ^2^ *d*_*i*_	*b*_*i*_	CV_*i*_	*θ*_(*i*)_	*θ*_*i*_	SR	AR	SD
MH1	6	10	10	8	7	10	5	7	7	7	6	6	6	5	7	6	6	119	7.000	1.572
MH2	4	1	1	1	1	1	1	1	1	1	1	1	1	3	1	1	11	32	1.882	2.423
MH3	2	9	9	6	5	6	3	4	4	4	8	8	8	8	5	8	4	101	5.941	2.182
MH4	9	6	8	11	11	6	11	10	11	10	10	10	9	11	11	10	2	156	9.176	2.382
MH5	8	4	6	4	6	6	7	5	5	5	3	3	3	1	4	3	9	82	4.824	1.977
MH6	5	11	11	10	8	11	5	8	8	8	11	11	11	10	9	11	1	149	8.765	2.755
MH7	11	2	3	9	9	4	10	9	10	9	7	7	7	7	8	7	5	124	7.294	2.468
MH8	1	4	4	2	2	4	4	3	2	3	5	5	5	4	2	5	7	62	3.647	1.493
MH9	3	6	5	3	3	2	2	2	3	1	2	2	2	9	6	2	10	63	3.706	2.538
MH10	7	8	7	5	4	3	8	6	6	5	4	4	4	2	3	4	8	88	5.176	1.855
MH11	10	2	2	7	10	9	9	11	9	10	9	9	10	6	10	9	3	135	7.941	2.838

Y: grain yield; SR: sum of rank; AR: average sum rank; SD: standard deviation.

**Table 4:** Estimation for sustainability index (SI) on grain yield of maize hybrids.

Genotypes	*Y*	*σn*	YM	SI (%)	
MH1	9.264	1.304	11.421	69.696	High
MH2	9.346	0.854	10.323	82.273	Very high
MH3	9.852	1.278	11.719	73.159	High
MH4	7.429	2.215	11.041	47.226	Moderate
MH5	8.510	1.072	10.385	71.620	High
MH6	9.316	1.743	11.944	63.401	High
MH7	6.959	1.261	8.076	70.558	High
MH8	9.904	1.060	11.083	79.804	High
MH9	9.480	1.272	11.064	74.191	High
MH10	8.745	1.071	9.859	77.833	High
MH11	7.107	1.703	9.807	55.101	Moderate

*Y*: mean yield; *σn*: standard deviation; YM: the best performance of a genotype in any environment; SI: sustainability index.

## Data Availability

The data used to support the findings of this study are included within the article.
